# Berberine Maintains the Neutrophil N1 Phenotype to Reverse Cancer Cell Resistance to Doxorubicin

**DOI:** 10.3389/fphar.2019.01658

**Published:** 2020-01-29

**Authors:** Shuhui Zhang, Lin Zhou, Mengdi Zhang, Yuehua Wang, Mengqi Wang, Jincheng Du, Wenwen Gu, Fuguang Kui, Jiahuan Li, Shengnan Geng, Gangjun Du

**Affiliations:** ^1^Institute of Pharmacy, Pharmaceutical College of Henan University, Kaifeng, China; ^2^School of Pharmacy and Chemical Engineering, Zhengzhou University of Industry Technology, Xinzheng, China; ^3^Chinese Medical School, Hunan University of Chinese Medicine, Changsha, China

**Keywords:** berberine, doxorubicin, neutrophil phenotype, carcinogenesis, chemotherapeutic resistance

## Abstract

This study explores the contributions of neutrophils to chemotherapeutic resistance and berberine-regulated cancer cell sensitivity to doxorubicin (DOX). *In vitro* experiments, continuous DOX treatment led to the shift of HL-60 cells to N2 neutrophils and thus induced chemotherapeutic resistance. The combination treatment with DOX and 2 µM berberine resulted in the differentiation of HL-60 cells toward N1 and therefore stimulated HL-60 cell immune clearance. Berberine increased reactive oxygen species (ROS) and decreased autophagy and therefore induced apoptosis in HL-60-N2 cells with morphological changes, but had no effect on cell viability in HL-60-N1 cells. The neutrophil-regulating efficacy of berberine was confirmed in the urethane-induced lung carcinogenic model and H22 liver cancer allograft model. Furthermore, we found that DOX-derived neutrophils had high levels of CD133 and CD309 surface expression, which prevented both chemotherapeutic sensitivity and immune rejection by self-expression of PD-L1 and surface expression of PD-1 receptor on T cells, whereas berberine could downregulate CD133 and CD309 surface expression. Finally, berberine-relevant targets and pathways were evaluated. This study first suggests an important role of berberine in regulating neutrophil phenotypes to maintain cancer cell sensitivity to DOX.

## Introduction

Cancer is a leading cause of human disease-related death, and chemotherapy is currently the standard of care (Chi et al., 2019; Matei et al., 2019). Cancer cells usually respond to initial chemotherapy but then become resistant and increase metastatic potential, which greatly contributes to mortality from most types of cancer (Berns and Berns, 2017; Wojtaszek et al., 2019). In this sense, cancer chemotherapy can stimulate tumor spread if cancer cells cannot be completely eliminated. Thus, it is crucial to elucidate the mechanisms underlying chemotherapeutic agent resistance in order to restore drug susceptibility in tumor cells. Previous studies of cancer chemotherapeutic resistance have focused on cancer cells themselves, including changes in apoptotic pathways, drug targets, ATP-binding cassette (ABC) transporter expression, and DNA damage repair (Kong et al., 2017; Wojtaszek et al., 2019). Although some chemotherapeutic sensitizers showed great promise in preclinical models, the currently available sensitizers have, disappointingly, not demonstrated complete or durable response rates in cancer patients (Fillmore et al., 2015; Thomas et al., 2018). Importantly, tumor cell persistence requires not only resistance to cell death but also immune escape in cancer bearing hosts (Hanahan and Weinberg, 2019; Ponzetta et al., 2019); however, the relationship between chemotherapeutic resistance and immune responses has received little attention.

Doxorubicin (DOX) is one of the most effective and widely used chemotherapeutic agents for both solid and hematologic tumors (Younes et al., 2014; Royer et al., 2016; Tap et al., 2016). Different from other chemotherapeutic agents that elicit nonimmunogenic apoptosis without an immunizing property, DOX treatment results in immunogenic cell death (ICD), which can elicit an effective anti-tumor immune response (Casares et al., 2005). Nevertheless, DOX, like other chemotherapeutic agents, also results in an immunosuppressive microenvironment that is favorable for tumor growth and progression, limiting and even removing cancer cell immune rejection (Amini et al., 2019). It is well known that both innate and adaptive immune responses play important roles in cancer progression and therapy (Karagiannis et al., 2017). Recently, neutrophils, the most important effectors of innate immunity, have been reported to have a crucial role in tumor initiation and progression (Nicolás-Ávila et al., 2017). In cancer patients, the intratumoral accumulation of tumor-infiltrated neutrophils (TINs) is positively correlated with poor prognosis (Wculek and Malanchi, 2015). Tumor-bearing animals also demonstrate a systemic increase in TINs, and TINs depletion increases tumor-infiltrating lymphocytes (TILs) and tumor response to other immunotherapies in preclinical studies (Coffelt et al., 2015). Whether DOX can induce TINs and whether these TINs are associated with tumor resistance remains poorly understood. Recent studies have shown that TINs are diverted to an immunosuppressive phenotype that stimulates Th2-type inflammation at the tumor site to support carcinogenesis and tumor progression (Uderhardt et al., 2019; Veglia et al., 2019). Berberine is an isoquinoline alkaloid from coptidis rhizomes and has anti-inflammatory properties (Zou et al., 2017). Here, we explored the contributions of neutrophils to DOX resistance and how berberine may regulate the sensitivity of cancer cells to DOX. Our results first indicated a vital role for neutrophil polarization in chemotherapeutic resistance and suggested a new mechanism by which the neutrophil to lymphocyte ratio (NLR) increases in cancer patients undergoing chemotherapy who have poor prognoses.

## Materials and Methods

### Materials

Berberine (purity > 98%, AB21379 was purchased from Lianshuo Biotechnology Co., Ltd. (Shanghai, China). DOX (D1515), urethane (U2500), all-trans retinoic acid (ATRA, PHR1187), TGF-β1 (616455), nitroblue tetrazolium (NBT, N6876), and 4′,6-diamidino-2-phenylindole (DAPI) (MBD0020) were purchased from Sigma Chemical Co (St. Louis. MO. USA). Anti-Ly6G microbeads (130-116-541) was from Miltenyi. Antibodies used included anti-CD66b (555723), anti-CD309 (550549), anti-CD133 (566595), anti-CD31 (562939), anti-P62 (611962), fluorescein isothiocyanate (FITC)-conjugated anti-mouse immunoglobulin G (IgG) (555988) were obtained from BD Pharmingen. Antibodies used included anti-STAT3 (60199-1-Ig), anti-PD-L1 (66248-1-Ig), anti-PD-1 (66220-1-Ig), β-actin (60008-1-Ig), anti-LC-3B (14600-1-AP), and anti-JAK2 (17670-1-AP) were obtained from Proteintech (Shanghai China). Horseradish peroxidase (HRP)-conjugated goat anti-mouse IgG polyclonal antibody (VC002), peroxidase substrate DAB (3, 3′-diaminobenzidine, 4800-30-07) were obtained from R&D Systems (Minnesota, USA). WP1066 (SD4749), dichloro-dihydro-fluorescein diacetate (DCFH-DA) (S0033) and were obtained from Beyotime (Shanghai China). Annexin V-FITC Apoptosis kit (CA1020) were obtained from Solarbio (Beijing China). Mouse quantitative ELISA kits, interferon (IFN)-γ (MIF00), interleukin (IL)-2 (M2000), IL10 (M1000B), tumor necrosis factor (TNF)-α (MTA00B), IL-6 (M6000B), TGF-β1 (MB100B), and PD-L1 (DY1019-05), were obtained from R&D Systems (Minnesota, USA). Standard rodent chow was purchased from Henan Provincial Medical Laboratory Animal Center (Zhengzhou, China), License No. SCXK (YU) 2015-0005, Certificate No. 41000100002406.

### Cell Culture and Assays

Human acute promyelocytic leukemia (HL-60) cells and mouse H22 hepatoma cells from American Type Culture Collection (ATCC) were purchased from the Chinese Academy of Sciences and were grown in RPMI 1640 medium supplemented with 10% (v/v) fetal bovine serum (FBS) in a humidified atmosphere containing 5% CO_2_ and 95% air at 37°C. To obtain N1-like neutrophils (N1), HL-60 cells were seeded at 2 × 10^5^ cells/ml in medium supplemented with 10 μM all-trans retinoic acid (named HL-60-N1) or 0.5 μM DOX (named HL-60-N1-D) for 7 days in a flask (Almzaiel et al., 2013; Li et al., 2018), changing the medium after 3 days. To obtain N2-like neutrophils (N2), HL-60-N1 cells were further stimulated with 100 ng/ml TGF-β1 for 3 days (Fridlender et al., 2009; Sagiv et al., 2015) and were named HL-60-N2. To collect cell-conditioned media, N1 or N2 cells were cultured in serum-free medium for 24 h, centrifuged to remove cells, further filtered to remove debris for supernatant collection, and named N1 cell-conditioned media (N1-CD) and N2 cell-conditioned media (N2-CD), respectively. The supernatant levels of IFN-γ, IL-2, PD-L1, IL-6, IL-10, and TGF-β1 were determined using ELISA kits according to the manufacturer's protocols. The results were calculated from linear curves obtained using the Quantikine kit standards.

For proliferation assays, HL-60 cells at 1 × 10^5^ cells/ml were seeded in a 96-well plate and treated with N1 or N2 cell-conditioned media, DOX or berberine alone or in combination for 48 h. N1 or N2 cells were also treated with DOX or berberine alone or in combination for 48 h, and living cells were examined by 3-(4,5-dimethylthiazol-2-yl)-2,5-diphenyltetrazolium bromide (MTT) reduction assay, according to our previous method (Liu et al., 2015). For differentiation analysis, HL-60 cells at 3 × 10^5^ cells/ml were seeded in six-well plates and treated with N1 or N2 cell-conditioned media, DOX or berberine alone or in combination for 5 days (changing the medium after 3 days), and neutrophil differentiation was assessed by Giemsa staining and microscopic NBT assay according to the previously described methods (Guo et al., 2017; Li et al., 2019). For the morphological assessment, cells were analyzed by a laser holographic cell imaging and analysis system (HoloMonitor M4, Phiab, Sweden). For phagocytic ability, intracellular phagocytosis of *Escherichia coli* was detected by Giemsa staining (Li et al., 2019). For autophagic analysis, cells were stained using FITC-conjugated anti-LC3-B or anti-p62 antibodies. For apoptotic analysis, the binding of ANXV-FITC to phosphatidylserine was measured by an automated cell counter and analysis system (Nexcelom Cellometer X2, Nexcelom, USA). For reactive oxygen species (ROS) measurement, the intracellular fluorescence of DCFH-DA was detected by a fluorescence spectrophotometer (Hitachi F-4600, Japan). For the time-lapse migration assay (Patel et al., 2018), cells were placed onto a motorized stage and observed with a laser holographic cell imaging and analysis system (HoloMonitor M4, Phiab, Sweden). A 20× objective was used to capture images during the course of the time-lapse. Images were captured every 15 s over the course of 30 min from at least four different fields of view.

Immunofluorescence was performed according to a previously described method (Guo et al., 2017). After overnight incubation with primary antibodies (CD66b, CD133, CD309, and PD-L1), slides were incubated with FITC-conjugated goat anti-mouse IgG for 30 min. The semi-quantitative immunofluorescence score was calculated by using the intensity score and proportion score by excluding the primary antibody and IgG matched serum as positive and negative controls, respectively.

### Western Blotting

HL-60-N1 and HL-60-N2 cells were treated with DOX or berberine alone or in combination in the presence or absence of WP1066 (a selective JAK2/STAT3 inhibitor) for 48 h. Proteins were extracted and separated *via* 12% sodium dodecyl sulfate-polyacrylamide gel electrophoresis, electroblotted onto nitrocellulose membranes, and probed with antibodies against CD66b, CD133, PD-L1, CD309, JAK2, and STAT3. Antibody binding was detected according to a previously described method (Guo et al., 2017).

### Hl-60 Cell Immune Clearance

HL-60 cell immune clearance was assessed using a calcein-release assay, according to our previously described method (Du et al., 2013). Briefly, CD8+ T cells were purified from ICR mouse spleens using the magnetic-activated cell sorting (MACS) separation system (Miltenyi Biotec, Bergisch Gladbach, Germany) and stimulated with phorbol 12-myristate 13-acetate (PMA) (10 ng/ml) and ionomycin (0.1 μg/ml) for 24 h in the presence of HL-60-N1 or HL-60-N2 or drug-treated HL-60 cell-conditioned media and harvested as the attacking cells. Mitomycin C-treated HL-60 cells were labeled with 10 μM calcein-AM as the target cells and placed into a 96-well plate with CD8+ T cells at ratios of 20:1, 10:1, and 5:1 (T cells: HL-60 cells) for 6 h at 37°C. The supernatants were transferred from each well to another 96-well plate, and fluorescence was measured using a Synergy2 multi-mode microplate reader (BioTek). Maximum release was obtained from detergent-released HL-60 cells, and spontaneous release was obtained from HL-60 cells incubated in the absence of CD8+ T cells (n = 5).

Immune clearance was determined as follows:

Immune clearance = (experimental release – spontaneous release) / (maximum release − spontaneous release) × 100%.

To detect how the different neutrophil phenotypes affect T lymphocytes, CD8+ T cells were cultured in the lower chamber at a concentration of 2 × 10^6^ cells/ml and were stimulated with PMA and ionomycin, and HL-60N1 or HL-60N2 cells were added to the upper chamber at a concentration of 2 × 10^6^ cells/ml in the presence or absence of anti-CD66b, anti-CD133, or anti-CD309 antibodies. After coincubation for 24 h at 37°C, the supernatant was centrifuged for the PD-L1 assay and CD8+ T cells in the lower chamber were collected for surface PD-1 receptor assay using immunohistochemistry according to previously described methods (Guo et al., 2017).

### Cytolytic Assay

The cytolytic activity of HL-60 cells was assessed by carboxyfluorescein succinimidyl ester (CFSE)-7AAD staining (Su et al., 2019). Briefly, HL-60 cells (target cells) were incubated with CFSE-labeled HL-60-N1 or HL-60-N2 cells or drug-treated HL-60 cells (attacking cells) at 10:1 and 5:1 (attacking cells: target cells) ratios for 6 h. Then, 7AAD was added to the cell suspensions and incubated on ice for 15 min. The percentages of 7AAD+ cells among CFSE+ cells were analyzed using an automated cell counter and analysis system.

### Animals

Ten-week-old female ICR mice were obtained from Henan Provincial Medical Laboratory Animal Center (Zhengzhou, China). All animal procedures were approved by the Animal Experimentation Ethics Committee of Henan University (permission number HUSAM 2016-288), and all procedures were performed in strict accordance with the Guide for the Care and Use of Laboratory Animals and the Regulation of Animal Protection Committee to minimize suffering and injury.

### Urethane-Induced Lung Carcinogenesis Model

Urethane (600 mg/kg body weight), alone or in combination with anti-Ly6G antibody (500 µg/mouse), was injected intraperitoneally (i.p.) into ICR mice once a week for 8 weeks, according to our previous protocol (Ma et al., 2016). Following the first urethane injection, mice received berberine (10 mg/kg) *via* intragastric administration once a day or DOX (5 mg/kg) *via* intravenous tail injection once a week alone or in combination for 12 weeks. At 13 weeks after the first urethane injection, orbital venous blood was collected for serum assays of PD-L1, IFN-γ, IL-2, TNF-α, IL-6, IL-10, and TGF-β1 using ELISA kits. Mice were sacrificed and cell-free alveolar fluid was collected by inserting a cannula into each trachea with three sequential injections of 1 ml phosphate-buffered saline (PBS), followed by centrifugation for cytokine assays (IFN-γ, IL-2, TNF-α, IL-6, IL-10, and TGF-β1), while the separated cells were resuspended in 0.9% sterile saline for total cell counts. Neutrophils in the suspensions were enriched by magnetic cell sorting utilizing anti-Ly6G-coated beads (providing >90% purity, as assessed by Wright-Giemsa staining), and neutrophil immunophenotypes were analyzed by FITC-conjugated anti-mouse CD66b, CD133, and CD309 (VEGFR2) staining. Neutrophil infiltration was observed in alveolar cavities using hemotoxylin and eosin (H&E) staining according to our previous methods (Liu et al., 2015; Li et al., 2019).

Spleen T lymphocytes (CD3+) were separated using the autoMACS separation system (Miltenyi Biotec, Bergisch Gladbach, Germany) for assays of cytotoxic CD8+ cell rates using an automated cell counter and analysis system.

Average numbers of lung carcinomas per mouse were calculated. A portion of each lung was preserved in 10% buffered formalin and routinely embedded in paraffin. Lung sections were stained for immunofluorescence according to our previous method (Guo et al., 2017). After overnight incubation with the primary antibodies (anti-mouse-CD31, anti-mouse-CD309, anti-mouse-tie2), slides were incubated with FITC-conjugated goat anti-mouse IgG for 30 min. The semi-quantitative immunofluorescence score was calculated. And spleen T lymphocyte surface PD-1 expression were analyzed by immunohistochemistry according to our previous method (Guo et al., 2017).

In addition, the lung vascular integrity was assayed with the Evans blue dye extra-barrier technique according to our previous method (Liu et al., 2015).

### Tumor Allograft Model

H22 cells were used for tumor allograft experiments. First, 200 µl saline containing 1 × 10^6^ cells was injected subcutaneously into the lateral axilla of mice to establish tumor allografts. One day after tumor inoculation, *in vitro* HL-60-derived HL-60-N1 or HL-60-N2 cells (2 × 10^6^ cells in 200 µl saline) were injected intravenously into mice once a week for 3 weeks; simultaneously, mice received berberine (10 mg/kg) *via* intragastric administration once a day, DOX (10 mg/kg) or anti-Ly6G antibody (500 µg/mouse) *via* tail intravenous injection once a week alone, or in combination for 3 weeks. Tumor size was monitored twice a week with callipers and calculated as the length×width2/2. On the 22nd day after tumor inoculation, orbital venous blood was collected for serum assays of PD-L1, IFN-γ, IL-2, TNF-α, IL-6, IL-10, and TGF-β1. Mice were euthanized, the tumors were extracted and weighed, bone marrow neutrophils were enriched by magnetic cell sorting utilizing anti-Ly6G-coated beads, and neutrophil immunophenotypes and spleen T lymphocyte surface PD-1 were analyzed by immunofluorescence. Spleen T lymphocytes were separated using the autoMACS separation system (Miltenyi Biotec, Bergisch Gladbach, Germany) for assays of cytotoxic CD8+ cell rate. The complete assay procedure was similar to methods in the urethane-induced lung carcinogenesis model.

In addition, the tumor vascular integrity was assayed with the Evans blue dye extra-barrier technique according to our previous method (Liu et al., 2015).

For the immune rechallenge study, the tails of 1/2 of the 60 mice were injected subcutaneously with 5 × 10^5^ H22 cells suspended in 50 μl saline. One day after tumor inoculation, the mice received berberine (10 mg/kg) *via* intragastric administration once a day, DOX (10 mg/kg) or anti-Ly6G antibody (500 µg/mouse) *via* tail intravenous injection once a week alone, or in combination for 2 weeks. Fifteen days after tumor implantation, the tumor-bearing tails were cut off to remove the primary tumors, and the mice were rechallenged with subcutaneous injections of 1 × 10^6^ H22 cells in 200 μl saline on their flanks. Tumor size was monitored twice a week with callipers. At 36 days, the same detections as above were carried out.

### The Regulatory Mechanism of Berberine on Neutrophils

The gene expression profiles GSE43254 and GSE101584 were obtained from the Gene Expression Omnibus (GEO) database (https://www.ncbi.nlm.nih.gov/geo ), and up- and downregulated genes related to tumor-associated neutrophils were identified using GEO2R, and the human structures of these differential proteins were collected from the protein data bank (PDB) for docking. The chemical structures of berberine and DOX were obtained from PubChem, and the docking exercise was conducted using the online software systemsDock (http://systemsdock.unit.oist.jp ) with the auto-removal of non-specified protein structures. Docking scores over 6 were regarded as potential targets for berberine and DOX. The gene ontology (GO) and Kyoto Encyclopedia of Genes and Genomes (KEGG) enrichment analyses were performed for the potential targets using the Database for Annotation, Visualization and Integrated Discovery (DAVID) (https://david.ncifcrf.gov/) and the online software ehbio (http://www.ehbio.com ). The compound-target-pathway network was constructed using Cytoscape3.2.1.

### Network Meta-Analysis

We systematically searched PubMed and Web of Science to identify eligible studies published from Jan 1, 2009 to Apr 1, 2019. The main terms “carcinoma,” “cancer,” “tumor,” and “chemotherapy” in the title as well as “neutrophil” and “lymphocyte” in the title/abstract, were used. Hazard ratios (HRs) with 95% confidence intervals (CIs) were used to detect the prognostic role of the NLR in chemotherapeutic cancer patients, focusing on overall survival (OS) and progression-free survival (PFS). Each included study was approved by an ethics committee or institutional review board. Exclusion criteria were: (1) no access to the full text for quality assessment and data extraction; (2) review articles; and (3) non-clinical studies or case reports. Fixed and random-effect meta-analyses were conducted based on the heterogeneity of the included studies.

### Statistical Analyses

The data were statistically analyzed using GraphPad Prism5.01 and presented as the mean ± SD. The differences between two groups were evaluated using a t-test. A P value of less than 0.05 was considered statistically significant. Meta-analyses were performed using using RevMan 5.3.

## Results

### Berberine Reverses the Doxorubicin-Stimulated Shift of HL-60 Cells to the HL-60-N2 Phenotype and the Chemotherapeutic Resistance of HL-60 Cells to Doxorubicin

Primary neutrophils are short-lived, limiting their experimental usefulness in the laboratory, and differentiated HL-60 cells are a valid model system for the analysis of human neutrophil behavior (Rincón et al., 2018) although the antimicrobial activities of HL-60 cells-differentiated neutrophil-like cells were distinctly lower compared to blood-derived neutrophils (Yaseen et al., 2017). To explore whether HL-60 cell-derived neutrophils also have similar properties to natural neutrophils, we induced the differentiation of HL-60 cells into N1-like neutrophils (HL-60-N1) and N2-like neutrophils (HL-60-N2), indicated by cytokine levels (**Supplementary Figures 1A–F**). As expected, compared to HL-60-N1 cells, HL-60-N2 cells had high levels of surface CD66b expression (**Figures 1A, B**) with morphological heterogenicity, as indicated by the cell distribution (**Figures 1C–E**). In bacterial phagocytosis, there was a significant difference between HL-60-N1 and HL-60-N2 cells (**Figure 1F**); simultaneously, HL-60-N2 cells had a reduction in ROS, as indicated by intracellular fluorescence of DCFH-DA (**Figure 1G**), and an increase in autophagy, as indicated by more LC3-B and the less p62 immunofluorescence (**Figure 2A**). When cocultured with HL-60N1 cell-conditioned media, HL-60 cells showed an increased apoptotic rate (**Figures 2B, C**) and a slowed proliferation rate, which were not affected by coculturing with HL-60-N2 cell-conditioned media (**Figure 2D**). Consistent with these results, HL-60-N1 cells led to HL-60 cell lysis, which was not influenced by HL-60-N2 cells (**Figure 2E**).

**Figure 1:** There is a difference between N1-like and N2-like neutrophils. N1-like and N2-like neutrophils were developed from the induced HL-60 cells. **(A**, **B)** Neutrophil CD66b expression was analyzed by fluorescein isothiocyanate (FITC)-conjugated anti-mouse CD66b staining (n = 5, 40×). **(C**, **D)** Neutrophil morphological changes analyzed by laser holographic cell imaging and analysis system (n = 5, 20×). **(E)** Neutrophil morphology indicated by Giemsa staining (n = 5, 100×). **(F)** Neutrophil phagocytosis detected by Giemsa staining (n = 5, 40×). **(G)** ROS detected by dichloro-dihydro-fluorescein diacetate (DCFH-DA) (n = 5). The data present mean ± SD, the experiments were repeated three times, and statistical significance was determined by a t-test. *P < 0.05, **P < 0.01 *vs.* HL60; ^#^P < 0.05, ^##^P < 0.01 *vs.* HL60-N2. DOX, doxorubicin; BER, berberine.

**Figure 2:** N1-like and N2-like neutrophils had different effects on HL-60 cells. **(A)** Cell autophagy as indicated by LC-3B and P62 staining (n = 5, 40×). **(B**, **C)** and **(C)** Cell apoptosis detected by the Annexin V-FITC apoptosis kit (n = 5). **(D)** HL-60 cell viability detected by 3-(4,5-dimethylthiazol-2-yl)-2,5-diphenyltetrazolium bromide (MTT) assay (n = 5). **(E)** Cytolytic activity (n = 5). The data present mean ± SD, the experiments were repeated three times, and statistical significance was determined by a t-test. **(A**, **C**, **D)** *P < 0.05, **P < 0.01 *vs.* HL60; ^##^P < 0.01 *vs.* HL60-N2. **(E)** *P < 0.05, **P < 0.01 *vs.* HL60-N1; ^##^P < 0.01 *vs.* HL60-N2. DOX, doxorubicin; BER, berberine.

To explore how neutrophil phenotype affect cancer cell chemotherapeutic resistance to DOX, we observed the effects of berberine and DOX on HL-60 cells and their differentiation. Expectedly, continuous DOX treatment led to HL-60 cell resistance to DOX (**Supplementary Figure 1G**) accompanied by the shift of HL-60 cells to the HL-60-N2 phenotype (**Figures 1A, B**). Unexpectedly, when administered at the dose (2 µM) that had little effect on cell viability in HL-60 and HL-60-N1 cells (**Supplementary Figure 1H**), berberine improved the morphological heterogenicity, as indicated by the cell distribution (**Figures 1C–E**) and ROS (**Figure 1G**), decreased autophagy (**Figure 2A**) and induced apoptosis in HL-60-N2 cells (**Figures 2B, C**), Importantly, the combination treatment with DOX and berberine resulted in the polarization of HL-60 cells toward the HL-60-N1 phenotype (**Figures 1A, B**), and these HL-60-N1 cells had the same roles as those induced by ATRA in HL-60 cell lysis (**Figure 2E**), and activated JAK2/STAT3 signaling (**Supplementary Figure 1I**).

### HL-60-N2 Cells Show a Stronger Stemness and Suppress CD8+ Cells

It is well known that a high NLR may be associated with an independently poor prognostic survival in cancer patients (Grenader et al., 2016), and to explore how neutrophils affect lymphocytes, we detected differences between N1-like and N2-like neutrophils and their influence on CD8+ T cells. Compared to HL-60-N1 cells, HL-60-N2 cells expressed stronger stemness, as indicated by CD133 and CD309 (**Figures 3A–C**), produced more PD-L1 (**Figures 3A, D**), and had higher mobility (**Figures 3E, F**) and JAK2/STAT3 inhibition (**Figure 3G**). DOX treatment caused cell differentiation and dispersion and increased these properties (**Figure 4A**), whereas berberine treatment alone or in combination with DOX resulted in cell differentiation but concentrated distribution and decreased these properties (**Figure 4A**). Cell function test showed that HL-60-N1 cell-conditioned media promoted immune clearance by CD8+ T cells compared to conditioned media from HL-60 cells, which was prevented by HL-60-N2 cell-conditioned media (**Figure 4B**). PD-1 and PD-L1 are immune checkpoint proteins whose binding ultimately result in T cell exhaustion and self-tolerance (Ancevski Hunter et al., 2018). PD-1 is mainly expressed on different immune cells, PD-L1 is regarded as the primary ligand of PD-1 (Pan et al., 2016). Recent studies have revealed that soluble PD-L1 (sPD-L1) in human cancers is potential diagnostic, therapeutic, or prognostic biomarker (Zhu and Lang, 2017). Considering the immunoregulatory effect of neutrophil-conditioned media, we believe that sPD-L1 has more biological significance than its membrane-bound form. Therefore, we examined the supernatant PDL-1 in N1-like and N2-like neutrophils and the surface PD-1 expression in CD8+ T cells. Consistent with function results, HL-60-N2 cells produced more PD-L1 (**Figure 4C**) and promoted CD8+ T cell expression of PD-1 surface receptor (**Figures 4D, E**). CD309 antibodies but not CD66b and CD133 antibodies prevented PD-L1 production in HL-60-N2 cells (**Figure 4C**) and PD-1 expression in CD8+ T cells (**Figures 4D, E**), whereas blocking JAK2/STAT3 signaling by WP1066 increased CD309 expression and PD-L1 production in HL-60-N2 cells (**Figure 4F**).

**Figure 3:** N1-like and N2-like neutrophils showed different phenotypic characteristics in stemness, mobility and jak2/stat3 signaling. **(A)** Cell protein expression of CD309, CD133, and PD-L1 indicated by immunofluorescence (n = 5, 40×). **(B**–**D)** Immunofluorescence score of **(A)** (n = 5). **(E)** Cell mobility observed by a laser holographic cell imaging and analysis system (n = 5, 20×). **(F)** The quantitative value of **(E)** (n = 5). **(G)** Protein expression levels of jak2/stat3 examined by Western blotting (n = 5). The data present mean ± SD, the experiments were repeated three times, and statistical significance was determined by a t-test. **(B**–**D**, **F)** *P < 0.05, **P < 0.01 *vs.* HL60; ^#^P < 0.05, ^##^P < 0.01 *vs.* HL60-N2. **(G)** *P < 0.05, **P < 0.01 *vs.* HL60-N2+BER; ^#^P < 0.05, ^##^P < 0.01 *vs.* HL60-N2. DOX, doxorubicin; BER, berberine.

**Figure 4:** The immunosuppression of N2-like neutrophils is associated with jak2/stat3 signal inhibition and the effect of the drug on HL-60-derived cells. **(A)** The effect of DOX and berberine on HL-60 cell differentiation (n = 5). **(B)** N1-like and N2-like neutrophils had different effects on CD8+ T cell immune clearance (n = 5). **(C)** PD-L1 production in HL-60 cell supernatant (n = 5). **(D**, **E)** PD-1 expression in CD8+ T cells examined by immunohistochemistry (n = 5, 40×). **(F)** and N2-like neutrophil protein expression examined by Western blotting (n = 5). The data present mean ± SD, the experiments were repeated three times, and statistical significance was determined by a t-test. **(A)** **P < 0.01 *vs*. HL60. (b).*P < 0.05, **P < 0.01 *vs*. control; **(C**, **D)** **P < 0.01 *vs*. HL60-N1; ^#^P < 0.05, ^##^P < 0.01 *vs*. HL60-N2. **(F)** *P < 0.05 *vs*. HL60-N2+BER; ^#^P < 0.05, ^##^P < 0.01 *vs*. HL60-N2. DOX, doxorubicin; BER, berberine.

### Berberine Maintains the Neutrophil N1 Phenotype to Reverse DOX-Promoted Carcinogenesis in a Urethane-Induced Lung Cancer Model

Immune surveillance plays a key role in carcinogenesis. To confirm the roles of neutrophils in carcinogenesis and DOX resistance, we investigated neutrophil phenotypes in a urethane-induced mouse lung cancer model. In this model, the tumor formation rate is 100% in control and DOX group (**Supplementary Figures 2A, B**), only one mouse died in DOX group during experiment. As expected, neutrophil infiltration in alveolar cavities was positively correlated with lung carcinogenesis in the control group, and both berberine treatment and neutrophil depletion induced by LY6G antibodies prevented lung carcinogenesis (**Figures 5A, B**, **Supplementary Figures 2A, B**). Unexpectedly, DOX alone promoted these incidents (**Figures 5A, B**, **Supplementary Figures 2A, B**). Immunophenotype assays showed that the infiltrated alveolar neutrophils were similar to HL-60-N2 cells and expressed more CD66b, CD133, and CD309 (**Figure 5C**) in the control group, indicating an N2 phenotype. ELISA results showed that the levels of Th1 cytokines (IFN-γ, IL-2, and TNF-α) decreased (**Supplementary Figures 2C–H**), and the levels of Th2 cytokines (IL-6, IL-10, and TGF-β1) increased (**Supplementary Figures 3A–C**, **Supplementary Figures 3D–F**) in serum and in alveolar cavities in control mice compared to levels in normal mice, indicating an immunosuppressive microenvironment during urethane carcinogenesis. This immunosuppressive microenvironment could be promoted by DOX and attenuated by berberine and therefore resulted in the more lung nodes in DOX group and the less lung nodes in berberine group than control. Importantly, the combination of DOX and berberine maintained the neutrophil N1 phenotype (**Figure 5C**) and decreased the NLR levels to reverse DOX-promoted carcinogenesis (**Figure 5D**), accompanied by a reduction in serum PD-L1 levels (**Figure 5E**), spleen T lymphocyte surface PD-1 expression (**Figure 5F**), lung tissue immunofluorescence staining of CD31, CD309, and tie2 (**Figure 5G**), permeability to Evans blue dye (**Figure 5H**), and increase in spleen cytotoxic CD8+ cell rates (**Figure 5I**), indicating a better restorage effect of berberine on anti-tumor immune response of DOX with the unchanged cancer cell sensitivity.

**Figure 5:** Neutrophils affect urethane-induced lung carcinogenesis. **(A)** Alveolar neutrophils indicated by hemotoxylin and eosin (H&E) staining of lung tissue (n = 5, 100×). **(B)** The number of lung nodes (n = 10). **(C)** Alveolar neutrophil protein expression of CD66b, CD309, and CD133 indicated by immunofluorescence (n = 5, 40×). **(D)** NLR in peripheral blood (n = 5). **(E)** Serum PD-L1 levels (n = 5). **(F)** Spleen tissue PD-1 expression examined by immunohistochemical analysis (n = 5, 100×). **(G)** Lung tissue protein expression of CD31, tie-2, and CD309 indicated by immunofluorescence (n = 5, 40×). **(H)** Lung tissue permeability to Evans blue (n = 5). **(I)** Spleen cytotoxic CD8+ cell rate (n = 5). The data present mean ± SD, the experiments were repeated three times, and statistical significance was determined by a t-test. *P < 0.05, **P < 0.01 *vs.* control. DOX, doxorubicin; BER, berberine.

### Berberine Maintains the Neutrophil N1 Phenotype to Promote Doxorubicin-Induced Tumor Suppression and to Reverse Doxorubicin-Induced Immunosuppression in the H22 Liver Cancer Allograft Model

To further confirm the roles of neutrophils in tumor progression and DOX resistance, we established an allograft model of H22 liver cancer and injected HL-60-N1 and HL-60-N2 cells *via* the tail vein into tumor-bearing mice. The HL-60-N2 cell injection promoted tumor growth, whereas the HL-60-N1 cell injection prevented tumor growth (**Figure 6A**), indicating a pro-tumor and anti-tumor function of neutrophils. Unlike the results in the urethane-induced lung cancer model, in this allograft model, berberine (10 mg/kg) or neutrophil depletion had a negligible effect on suppression of tumor growth, while DOX significantly suppressed tumor growth (**Figure 6A**). The tumor-suppressing efficacy of DOX was promoted by berberine, neutrophil depletion, and HL-60-N1 cell injection, which decreased the NLR levels (**Figure 6B**) and the intratumor permeability to Evans blue dye (**Figure 6C**), but was attenuated by HL-60-N2 cell injection, which increased the intratumor permeability to Evans blue dye (**Figure 6C**). The results of bone marrow neutrophil immunophenotypes (**Figure 6D**), serum cytokines (**Supplementary Figures 4A–F**), and spleen T lymphocytes (**Figure 6E**) were similar to those in the urethane-induced lung cancer model, indicating a N2 neutrophil-polarizing efficacy of DOX. The immunosuppressive efficacy of DOX-induced neutrophils was further confirmed in a H22 cell rechallenge immune study where tumor immune rejection was suppressed by DOX but was promoted by berberine (**Figure 6F**). Importantly, the combination of DOX and berberine synergistically stimulated H22 cell immune rejection accompanied by a reduction in bone marrow N2 neutrophils (**Figure 6G**) intratumor permeability to Evans blue dye (**Figure 6H**), NLR levels (**Figure 6I**), serum levels of PD-L1 (**Figure 6J**), Th2 cytokines (**Supplementary Figures 5D–F**), and spleen T lymphocyte surface PD-1 expression (**Figure 6K**). Conversely, this combination increased bone marrow N1 neutrophils (**Figure 6G**), serum Th1 cytokines (**Supplementary Figures 5A–C**), and spleen memory CD8+ cell rates (CD8+CD45RA− cells) (**Figure 6L**), indicating a maintenance effect of berberine on the N1 neutrophil phenotype. The immune-rejecting efficacy of berberine on tumor rechallenge could be abrogated by neutrophil depletion, indicating an important role of neutrophils in secondary immunity and immune memory. It is worth mentioning that the expression of CD66b and CD309 of the combination of berberine and anti-Ly6G was higher than berberine or anti-Ly6G alone while anti-Ly6G and berberine could lower the expression of CD66b and CD309, indicating an interaction elimination effect between berberine and anti-Ly6G and a N2 neutrophil repolarization but not dual suppressive action of the combination of berberine and anti-Ly6G.

**Figure 6:** N2-like neutrophils are related to tumor sensitivity to DOX and tumor secondary immunity and immune memory. **(A)** Tumor weight (n = 6). **(B)** Tumor tissue permeability to Evans blue (n = 6). **(C)** Neutrophil to lymphocyte ratio (NLR) in peripheral blood in tumor-bearing mice (n = 6). **(D)** Bone marrow neutrophil immunophenotypes indicated by immunofluorescence (n = 6, 40×). **(E)** Spleen cytotoxic CD8+ cell rate (n = 6, 40×). **(F)** Tumor growth curve in a tumor rechallenge immune study. (n = 6). **(G)** Bone marrow neutrophil immunophenotypes indicated by immunofluorescence (n = 6, 40×). **(H)** Tumor tissue permeability to Evans blue (n = 6). **(I)** NLR in peripheral blood (n = 6). **(J)** Serum PD-L1 levels (n = 6). **(K)** Spleen tissue PD-1 expression indicated by immunofluorescence. (n = 5, 40×). **(L)** Spleen memory CD8+ cell rate (n = 6). The data present mean ± SD, the experiments were repeated three times, and statistical significance was determined by a t-test. *P < 0.05, **P < 0.01 *vs.* control; ^#^P < 0.05, ^##^P < 0.01 *vs.* DOX. DOX, doxorubicin; BER, berberine.

### Berberine Maintains the Neutrophil N1 Phenotype by Targeting the Multiprotein Network

We queried 858 upregulated genes (LogFC ≥ 1.5, P < 0.05) and 1,033 downregulated genes (LogFC ≤ -1.5, P < 0.05) related to tumor-associated neutrophils and obtained targeting information on 357 genes. A total of 165 potential targets with docking scores >6.0 (pKd/pKi) associated with DOX and berberine were selected for GO and KEGG analyses. KEGG enrichment analysis revealed that the berberine-associated reversal of potential targets of DOX to regulate neutrophils was significantly enriched in the “pathways in cancer,” “JAK-STAT signaling pathway,” and “FoxO signaling pathways” terms (**Figure 7A**, **Supplementary Figure 6**). GO enrichment analysis indicated that the berberine-associated reversal of the potential targets of DOX to regulate neutrophils was primarily associated with the “innate immune response,” “apoptotic process,” and “oxidation−reduction process” terms (**Supplementary Figure 7**).

**Figure 7:** The potential targets of DOX and berberine in regulating neutrophils analyzed by network pharmacology and a predictive role of neutrophil to lymphocyte ratio (NLR) in chemotherapy sensitivity of cancer patients. **(A)** The potential targets of DOX and berberine in regulating neutrophils. **(B)** Effect of NLR on progression-free survival (PFS) in cancer patients receiving chemotherapy in the meta-analysis shown as the forest map and the funnel diagram. **(C)** Effect of NLR on OS in cancer patients receiving chemotherapy in the meta-analysis shown as the forest map and the funnel diagram. **(D)** Effect of NLR on overall survival (OS) in cancer patients receiving combination chemotherapy in the meta-analysis shown as the forest map and the funnel diagram. **(E)** Effect of NLR on adverse effects in cancer patients receiving chemotherapy in the meta-analysis shown as the forest map and the funnel diagram. DOX, doxorubicin.

### The Neutrophil to Lymphocyte Ratio Is Adversely Prognostic in Chemotherapeutic Drug-Treated Cancer Patents

A total of 26 observational clinical articles (7 prospective studies and 19 retrospective studies) including 7,907 patients were included in the meta-analysis. Pretreatment or post-treatment with higher NLRs than the median had significant impacts on PFS (HR = 1.63, 95% CI:1.55-1.72; P = 0.00001) (**Figure 7B**) and OS (HR = 1.54, 95% CI: 1.48–1.61; P = 0.00001) in cancer patients undergoing chemotherapy (**Figure 7C**). No significant difference was presented in the sensitivity analysis. According to the five articles concerning combination chemotherapy that included 2,651 participants, we found that the post-treatment reduction in NLRs significantly improved OS (HR = 1.81, 95% CI: 1.68–1.96; P = 0.00001) (**Figure 7D**). Meanwhile, patients with lower baseline NLR underwent less adverse effects (RR = 1.24, 95% CI: 1.18–1.3; P = 0.00001) (**Figure 7E**), indicating a predictive role of NLRs in chemotherapy sensitivity of cancer patients.

## Discussion

Neutrophils are important first responders known as cells of the innate immune system traffic to sites of infection and injury and play diverse and critical roles in the removal of necrotic cell debris for tissue repair and inflammation resolution. There are many necrotic cells in tumors due to rapid proliferation-related hypoxia (Daniels et al., 2017). Systemic cancer chemotherapy exerts extensive cytotoxic effects and results in immunogenic or nonimmunogenic cell death of tumor and normal tissue (Verwaal et al., 2003; Kono et al., 2013; Kuijpers et al., 2014). These excessive dead cells are beyond the scavenging capacity of professional and non-professional neighboring phagocytes and are able to mimic pathogen response-like recruitment of neutrophils to maintain unresolved inflammation for cancer initiation and progression (Garg et al., 2017). However, the nature and function of TINs only recently began to be unveiled, and the greater contribution of neutrophils to cancer development must be investigated. Eruslanov EB et al. found that TINs could stimulate T cell responses in early-stage human lung cancer, indicating an immunostimulative function of neutrophils in the earliest stages of cancer, although neutrophils are one of the most important immunosuppressors (Eruslanov et al., 2014). In this study, we first showed that continuous DOX treatment promoted the shift of HL-60 cells or TINs to N2-type neutrophils and thus induced chemotherapeutic resistance, indicating a new function of neutrophils in cancer chemotherapeutic resistance.

Neutrophils possess functional plasticity, and their subsets have distinct phenotypic characteristics (N1 or N2) and can exhibit both pro- or antitumorigenic properties, depending on their phenotype (Riffelmacher et al., 2017). N1 is a mature and homogenous population of high-density neutrophils that can acquire a cytotoxic phenotype to exert anti-tumor functions in response to a variety of stimuli. In contrast, N2 is a heterogeneous population of low-density neutrophils that display pro-inflammatory and immunosuppressive properties to exert pro-tumor functions (Sagiv et al., 2015; Riffelmacher et al., 2017). In cancer patients, neutrophils, like other myeloid cells, are kept in an immature state of differentiation, rather than the anti-tumor N1 or pro-tumor N2 phenotype (Ponzetta et al., 2019). Consistent with these previous reports, in this study, we found that TINs showed a classic CD66b+ N2 phenotype and simultaneously expressed the stemness markers CD133 and CD309, indicating an immature phenotype. Unexpectedly, TINs could be further polarized by DOX toward the N2 phenotype and therefore prevented both chemotherapeutic sensitivity and the tumor immune rejection by apoptotic induction of cytotoxic T lymphocytes, which can explain why tumor chemotherapy and immunotherapy have synergistic therapeutic effects and why the NLR is an independent prognostic factor in cancer patients. Certainly, in the strict sense, the N2 type neutrophil ratio should be used for predicting treatment outcome in cancer. We found that berberine could selectively impact N2-type neutrophils to maintain the N1 neutrophil phenotype, thus preventing TINs polarization to the N2 phenotype and reversing tumor resistance to DOX. The meta-analysis showed that the NLR is highly prognostic across many tumor types in cancer patients undergoing chemotherapy, suggesting a wide role of neutrophils in chemotherapeutic resistance. A mechanistic understanding of the role of TINs in tumor progression and chemotherapeutic resistance will provide unique therapeutic alternatives.

Chemotherapy plays a crucial role in controlling tumor progression; however, an increasing number of studies have indicated that subsequent tumor regression depends on sustained Th1 immune responses after cancer chemotherapy (Böhm et al., 2016; Kaewkangsadan et al., 2016). Therefore, the immunogenic cell death induced by a specific set of chemotherapeutic drugs is expected. In previous studies, tumor cells dying in response to DOX can elicit an effective anti-tumor immune response in the absence of any adjuvant (Du et al., 2010). These experiments did not take into account the long-term interaction of chemotherapy with the immune system. In fact, most patients became resistant to DOX and immune suppression soon after repeated treatment (Royer et al., 2016). This suggests that the chemotherapy-induced tumor immune response cannot eliminate tumor cells and even promotes immune tolerance. In this study, we found that continuous DOX treatment suppressed tumor immune rejection, which could be synergistically stimulated by the combination of DOX and berberine, whereas neutrophil depletion led to abrogation of the combined immune-rejecting efficacy. It was also previously reported that immunosuppressive neutrophils decreased human leukocyte antigen (HLA)-DR expression to reduce the switch to the adaptive response (Pollyea et al., 2018). Based on these results, we believe that neutrophil phenotypes may determine the immunosuppressive or immunosurveillance microenvironment and therefore affect tumor responses to chemotherapy.

Berberine is extracted from Rhizoma Coptis (Huanglian in Chinese), which has been extensively used for treating infectious diarrhea, heat-clearing, and detoxifying for thousands of years in traditional Chinese medicine. Previous studies demonstrated that berberine possesses various pharmacological activities and may treat different diseases, such as sepsis, inflammation, diabetes and cancer, by multiple mechanisms, e.g., halting cell cycle progression and triggering apoptosis (Chen et al., 2017; Hou et al., 2017; Zou et al., 2017). In cancer cells, berberine could induce apoptosis and inhibit the chemotherapy-induced repopulation by suppressing the arachidonic acid metabolic pathway (Li et al., 2015; Zhao et al., 2017), enhance chemosensitivity through dose-orchestrated AMPK signaling (Pan et al., 2017), and reverses hypoxia-induced chemoresistance through the inhibition of AMPK-HIF-1α (Pan et al., 2017), In addition, berberine also plays a role in the regulation of immune response, oxidant stress, tissue fibrosis, and autophagy with low side effects and good resistance, suggesting its clinical and research values (Yang et al., 2019). In this study, berberine alone or in combination with doxorubicin maintained the N1 neutrophil phenotype to prevent carcinogenesis and chemotherapeutic resistance. Bioinformatics analysis found that the potential targets of berberine regulation of neutrophils were primarily associated with the “innate immune response,” “apoptotic process,” and “oxidation−reduction process,” indicating a function of berberine targeting the multiprotein network, such as “pathways in cancer,” “Jak-STAT signaling pathway,” and “FoxO signaling pathways,” whereby berberine regulates neutrophil phenotypes to maintain immune surveillance and cancer cell sensitivity to DOX. We used a pharmacological blocker to confirm the important role of JAK-STAT signaling in berberine-regulated neutrophil functions, and found that CD309 antibodies prevented production of PD-L1 by N2-like neutrophils and PD-1 expression by CD8+ T cells, whereas blocking JAK/STAT3 signaling increased CD309 expression by N2-like neutrophil, indicating an association between N2 neutrophil functions and the JAK/STAT3-CD309-PD-L1 feedback loop. Certainly, this is only one of the important feedback loops.

In summary, tumor- and chemotherapy-induced N2-type neutrophils play a crucial role in cancer cell resistance to DOX, and our findings suggest several potential clinical implications. First, N2 neutrophil accumulation correlates with cancer progression and cancer cell resistance to chemotherapy, supporting TINs as a therapeutic target to promote DOX-based chemosensitivity. Second, alteration of the neutrophil phenotype is superior to depletion of TINs for reversing chemoresistance and immune escape, indicating the potential of re-educating these cells to reverse their pro-tumor functions for anti-tumor properties. Third, neutrophils, as the first responders of innate immune surveillance, can not only enhance tumor cell susceptibility to chemotherapy but also restore the function of exhausted T cells, providing a novel strategy for resolving the contradiction between chemotherapy-induced immunological cytotoxicity and immune system-induced tumor rejection. Certainly, whether re-educating TINs is the most effective approach for reversing the immunosuppressive environment needs to be fully evaluated.

## Data Availability Statement

All datasets generated for this study are included in the article/**Supplementary Material**.

## Ethics Statement

The animal study was reviewed and approved by the Animal Experimentation Ethics Committee of Henan University.

## Author Contributions

Conceived and designed the experiments: GD. Performed the experiments: SZ, LZ, MZ, YW, MW, JD, WG, FK, SG. Analyzed the data: GD, SZ, JL, SG. Contributed reagents/materials/analysis tools: GD. Wrote the paper and plotted the results: GD, SZ, LZ.

## Funding

Natural Science Foundation of Henan Province (No. 182300410310). Postgraduate Education Reform Project of Henan Province (No. hnyjs2015kc24). Postgraduate Education Innovation and Quality Improvement Project of Henan University (No. SYL18060136, SYL18060137, SYL19060140 and SYL19060139).

## Conflict of Interest

The authors declare that the research was conducted in the absence of any commercial or financial relationships that could be construed as a potential conflict of interest.

## Supplementary Material

Supplementary Figure 1 (a), (b), (c), (d), (e) and (f) Supernatant cytokine levels in cell culture (n = 5). (g) DOX induced HL-60 cell resistance (n = 5). (h) Berberine had an effect on cell viability in HL-60 and N2-like neutrophils (n = 5). (i) Protein expression examined by Western blotting (n = 5). The data present Mean ± SD, the experiments were repeated 3 times, and statistical significance was determined by a t-test. *P < 0.05, **P < 0.01 vs HL60, (g) *P < 0.05, **P < 0.01 vs WT-HL60. DOX: Doxorubicin, BER: Berberine.

Supplementary Figure 2 (a): Urethane-induced lung appearance (n = 10) and H&E staining of lung tissue (n = 5, 100×). (b) The tumor formation rate (n = 10). (c), (d), (e), Serum cytokine levels in urethane-induced lung cancer mice (n = 5). (f), (g) and (h) Alveolar cytokine levels in urethane-induced lung cancer mice (n = 5). The data present Mean ± SD, the experiments were repeated 3 times, and statistical significance was determined by a t-test. (b) *P < 0.05, **P < 0.01 vs control. (c), (d), (e), (f), (g) and (h) *P < 0.05, **P < 0.01 vs normal; #P < 0.05, ##P < 0.01 vs control. DOX: Doxorubicin, BER: Berberine.

Supplementary Figure 3 (a), (b) and (c) Serum cytokine levels in urethane-induced lung cancer mice (n = 5). (d), (e) and (f) Alveolar cytokine levels in urethane-induced lung cancer mice (n = 5). The data present Mean ± SD, the experiments were repeated 3 times, and statistical significance was determined by a t-test. *P < 0.05, **P < 0.01 vs normal; #P < 0.05, ##P < 0.01 vs control. DOX: Doxorubicin, BER: Berberine.

Supplementary Figure 4 Serum cytokine levels in tumour allograft. (n = 6). The data present Mean ± SD, the experiments were repeated 3 times, and statistical significance was determined by a t-test. *P < 0.05, **P < 0.01 vs control. DOX: Doxorubicin, BER: Berberine.

Supplementary Figure 5 Serum Th1 cytokines and Th2 cytokines in tumor rechallenge immune study (n = 6). The data present Mean ± SD, the experiments were repeated 3 times, and statistical significance was determined by a t-test. *P < 0.05, **P < 0.01 vs control. DOX: Doxorubicin, BER: Berberine.

Supplementary Figure 6 KEGG enrichment analysis performed by DAVID and visualized by ehbio.

Supplementary Figure 7 GO enrichment analysis performed by DAVID and visualized by ehbio.
